This article has been retracted.

# Propofol inhibits oxidative stress injury through the glycogen synthase kinase 3 beta/nuclear factor erythroid 2-related factor 2/heme oxygenase-1 signaling pathway

**DOI:** 10.1080/21655979.2021.2021062

**Published:** 2022-01-14

**Authors:** Ziyin Zhang, BaoFeng Yan, Yuguo Li, Shuo Yang, Jinfeng Li

**Affiliations:** a Department of Anesthesiology, The First Affiliated Hospital of Guangzhou University of Chinese Medicine, Guangdong, China; b Department of Anesthesiology, Fifth Medical Center of Chinese Pla General Hospital, Beijing, China; c Department of Anesthesiology, The Second Affiliated Hospital of Guangzhou University of Chinese Medicine, Guangdong, China; d Department of Medical Administration, The Eleventh People’s Hospital of Guangzhou, Guangdong, China

**Keywords:** Propofol, cardiomyocyte injury, oxidative stress, myocardial ischemic reperfusion injury (MIRI), GSK3β-Nrf2/HO-1

## Abstract

Oxidative stress is the main cause of ischemia/reperfusion injury. Propofol is a commonly used intravenous hypnotic anesthetic agent with antioxidant properties. In this study, we aimed to elucidate the protective effects of propofol on H_2_O_2_-induced cardiomyocyte injury and myocardial ischemic/reperfusion injury (MIRI) in rats. Cardiomyocyte injury was evaluated by determining cardiac troponin-1 (cTn-1) and creatine kinase-MB (CK-MB) levels. Antioxidative stress was assessed by measuring lactate dehydrogenase (LDH), malondialdehyde (MDA), glutathione (GSH), superoxide dismutase (SOD), reactive oxygen species (ROS), and catalase (CAT) levels. Apoptosis was evaluated using flow cytometry and TUNEL assays. Bax and Bcl-2 expression levels were determined by quantitative reverse transcription PCR (qRT-PCR) and Western blotting. The levels of glycogen synthase kinase 3 beta/nuclear factor erythroid 2-related factor 2 (Nrf2)/heme oxygenase-1 (HO-1) pathway-related factors were measured using Western blotting. Myocardial infarction in rats was analyzed using an Evans blue staining assay. The results showed that propofol reduced the levels of CK-MB, cTn-1, LDH, MDA, and ROS, and increased the levels of GSH, SOD, and CAT in H_2_O_2_-treated H9c2 cells. Additionally, propofol inhibited H_2_O_2_-induced apoptosis by downregulating Bax and upregulating Bcl-2. Moreover, propofol decreased the area of myocardial infarction in rats with MIRI. The GSK3β-Nrf2/HO-1 signaling pathway was activated by propofol. Rescue experiments showed that Nrf2 knockdown alleviated the effects of propofol on oxidative stress and apoptosis in H9c2 cells. In conclusion, propofol attenuated H_2_O_2_-induced myocardial cell injury by regulating the GSK3β/Nrf2/HO-1 signaling pathway and alleviating MIRI, suggesting that propofol is a promising therapeutic option for ischemic heart disease.

## 1. Introduction

Ischemic heart disease has high morbidity and mortality rates and imparts a large burden on public health globally [1]. Recently, preserving a viable myocardium by restoring normal blood flow or by pharmacological means, has become an effective myocardial infraction treatment strategy [2]. A reduction in myocardial damage has been observed during reperfusion, but this process itself can promote localized oxidative stress and a regional inflammatory reaction, causing cellular damage and, in some cases, death [3]. This pathophysiological process is known as myocardial ischemia/reperfusion injury (MIRI) [4]. The underlying mechanism of MIRI is intricate and involves complex signaling networks.

Activation of the phosphoinositide 3-kinase (PI3K)/protein kinase B (AKT)/glycogen synthase kinase 3 beta (GSK3β)-dependent signaling pathway can alleviate MIRI [5]. *GSK3β* is a downstream gene of the PI3K/AKT pathway and it regulates multiple cellular processes, such as signal transduction, metabolism, cell survival, and cell death [6]. Inactivation of GSK3β by phosphorylation induces nuclear factor erythroid 2-related factor 2 (Nrf2) nuclear translocation to protect cells from oxidative stress [7]. Nrf2 is important for maintaining redox homeostasis and regulating antioxidant response elements, including heme oxygenase-1 (HO-1) [8]. Nrf2/HO-1 are proteins that are present in all cells. When activated, Nrf2 is transferred to the nucleus where it binds to DNA through HO-1, thus regulating oxidative stress, ferroptosis, pyroptosis, and autophagy [9]. The GSK3β-Nrf2/HO-1 pathway is also critically involved in cardiovascular diseases, including MIRI [10,11]. However, the effect of this pathway on MIRI remains unclear.

There are currently various treatments used for MIRI [12]. Propofol is a rapid, short-acting intravenous hypnotic anesthetic agent commonly used during and after cardiac operations [13,14]. Propofol is also used to treat various other diseases, such as cancer, cardiac disease, and Parkinson’s disease [15–17]. Previous reports have distinctly shown the protective effect of propofol against MIRI [18,19]. Furthermore, the effect of propofol is mediated through various signaling pathways, such as the MAPK/ERK and JAK/STAT pathways [20,21]. However, since propofol has antioxidant properties, its effects on the GSK3β-Nrf2/HO-1 pathway in MIRI require further investigation.

Accordingly, we aimed to elucidate the effect of propofol on H_2_O_2_-treated myocardial cells and rats with MIRI. We hypothesized that propofol inhibits myocardial damage, oxidative stress, and apoptosis of H_2_O_2_-treated H9c2 cells, and decreases the incidence of myocardial infarction in rats with MIRI. Moreover, the effect of propofol on regulating the GSK3β-Nrf2/HO-1 signaling pathway was determined. The goal of this study was to provide new insights into the treatment of ischemic heart disease.

## 2. Materials and methods

### 2.1. Cell culture

Rat H9c2 cells were obtained from the Cell Bank of the Chinese Academy of Sciences (Shanghai, China). Cells were cultured in Dulbecco’s modified Eagle’s medium (Invitrogen, Carlsbad, CA, USA) supplemented with 10% fetal bovine serum (Invitrogen) in a humidified incubator at 37°C and 5% CO_2_. When the cells reached 70–80% confluence, they were digested with 0.25% trypsin for further analysis.

### 2.2. In vitro *experimental protocol*

H9c2 cells were divided into the following four groups: control (CON), H_2_O_2_, low-dose propofol (L-PRO), and high-dose propofol (H-PRO) groups. Cells in the H_2_O_2_ group were cultured with 100 μM H_2_O_2_ for 24 h, cells in the L-PRO group were cultured with 100 μM H_2_O_2_ and 50 μM propofol for 24 h, and cells in the H-PRO group were cultured with 100 μM H_2_O_2_ and 100 μM propofol for 24 h.

### 2.3. Cell counting kit-8 assay

H9c2 cells were seeded in 96-well plates and treated with 0, 50, 100, or 200 μM propofol for 24 h. Subsequently, the cells were incubated with 10 μL of Cell Counting Kit-8 solution (DOJINDO, Kumamoto, Japan) at 37°C for 4 h. Finally, the optical density was measured at 450 nm using a microplate reader (Bio-Tek, Winooski, VT, USA).

### 2.4. Cell transfection

A short hairpin (sh) RNA negative control (sh-NC) and sh-*Nrf2* were purchased from GenePharma (Shanghai, China). Cells in the H-PRO group were seeded into 6-well plates and transfected with sh-NC and sh-Nrf2 using Lipofectamine 2000 reagent (Invitrogen) following the manufacturer’s protocol. After 48 h, the expression level of Nrf2 was detected by quantitative reverse transcription PCR (qRT-PCR).

### 2.3. Apoptosis analysis

Flow cytometry was performed as described previously [22]. H9c2 cells were stained with propidium iodide/annexin V-FITC apoptosis kit (Beyotime, Shanghai, China) and analyzed using a BD FACSVerse flow cytometer (BD Biosciences, Franklin Lakes, NJ, USA) following the manufacturer’s protocols.

### 2.4. TUNEL staining

The TUNEL assay was performed as previously described [23]. H9c2 cells in each group were cultured in 6-well plates until the cells covered more than 70% of the wells. The cells were then fixed with 4% formaldehyde for 15 min and dehydrated with 50%, 75%, 95%, and 100% ethanol for 5 min each. The cells were then washed twice with phosphate buffer solution and treated with 0.5% Triton X-100 for 20 min. Finally, the TUNEL working solution was added and the cells were incubated at 37°C for 1 h.

### 2.5. Determination of cardiac troponin-1, creatine kinase-MB, lactate dehydrogenase, malondialdehyde, glutathione, superoxide dismutase, and catalase levels

The supernatants of cultured cells in each group were used to measure the levels of creatine kinase-MB (CK-MB) and cardiac troponin-1 (cTn-1) using an enzyme-linked immunosorbent assay (ELISA; R&D Systems, Minneapolis, MN, USA) [24] and to determine lactate dehydrogenase (LDH), glutathione (GSH), superoxide dismutase (SOD), malondialdehyde (MDA), and catalase (CAT) levels using corresponding kits (Nanjing Jiancheng Bioengineering, Inc., Nanjing, China), according to the manufacturer’s protocols.

### 2.6. Determination of reactive oxygen species

After the cells were treated with propofol and transfected with shRNAs, they were preloaded with 10 μM 2ʹ-7ʹ-dichlorofluorescein diacetate (Beyotime) for 20 min. After washing with serum-free medium, the intensity of dichlorofluorescein fluorescence was measured using a fluorescence microplate reader [25].

### 2.7. qRT-PCR

TRIzol (Shanghai Pufei Biotech Co., Ltd., Shanghai, China) was used to extract and purify total RNA from cells according to the manufacturer’s instructions. Gene expression levels were determined using the SYBR Master Mix Kit (TAKARA, Kusatsu, Japan) on a LightCycler480 qRT-PCR platform (Roche, Basel, Switzerland). The following cycling conditions were used: 95°C for 30 s; 40 cycles of 95°C for 5 s and 60°C for 30 s. mRNA expression levels were calculated using the 2^−ΔΔCT^ method. *GAPDH* was used as the internal standard.

### 2.8. Western blotting

Protein samples were extracted from tissues of each group, separated by sodium dodecyl sulfate-polyacrylamide gel electrophoresis, and transferred onto polyvinylidene fluoride membranes. After transfer, the membranes were blocked with 5% nonfat milk at room temperature for 1 hour. The membranes were then probed with specific antibodies against the target proteins and incubated at 4°C overnight. The primary antibodies included anti-Nrf2, anti-HO-1, anti-Bcl-2, anti-Bax, anti-p-GSK3β, and anti-GSK3β antibodies (all 1:1,000; Abcam, Cambridge, UK). The next day, the membranes were washed three times and then incubated with secondary antibodies (1:2,000, Abcam). Finally, the membranes were washed thrice. Protein expression levels were visualized using a chemiluminescence reagent and analyzed using ImageJ software (National Institutes of Health, Bethesda, MD, USA).

### 2.9. Animal experiments

Healthy male Sprague-Dawley rats weighing 230–260 g were supplied by the Animal Center of Guangzhou University of Traditional Chinese Medicine. All animals were maintained in accordance with the guidelines of use and care published by the Second Affiliated Hospital of Guangzhou University of Chinese Medicine.

Rats were divided into the following four groups: sham, MIRI, MIRI + L-PRO, and MIRI + H-PRO. A total of eight rats per group. Two rats failed to establish the MIRI model or died. Thus, each group contained 5 rats. The rats were anesthetized with 10% chloral hydrate (330 mg/kg) by injection into the gluteus maximus muscle and were artificially ventilated using a rodent ventilator. The rats’ respiration rate was synchronized spontaneously at 70 strokes/min (tidal volume: 20 mL). Surgery was performed on the rats by inducing a left thoracotomy opening, followed by pericardiotomy. Sutures were then passed around the left anterior descending (LAD) coronary artery, and a snare was formed by tightly pulling the artery’s ends around a small vinyl tube. Epicardial cyanosis was used to confirm coronary artery occlusion. Ischemia was maintained for 30 min, followed by myocardial reperfusion for 2 h. The snare was released to achieve successful reperfusion, as confirmed by epicardial hyperemia.

In the MIRI + L-PRO and MIRI + H-PRO groups, propofol was injected intraperitoneally for 7 days before reperfusion. In the sham and MIRI groups, the rats were separately injected with equal volumes of saline.

After reperfusion, the LAD coronary artery was occluded and injected with 2 mL of 1% Evans blue dye through the femoral vein to distinguish between perfused and non-perfused sections of the heart. The Evans blue solution stains the perfused myocardium, while the occluded vascular bed remains unstained. The following formula was used to determine the infraction size: infarct area/area at risk × 100%.

### 2.10. Statistical analysis

All data are expressed as the mean ± standard deviation. Statistical analyses were performed using Prism 6 software (GraphPad, San Diego, CA, USA). One-way analysis of variance was used to compare the different groups, followed by Tukey’s test. Statistical significance was set at *P* < 0.05.

## 3. Results

In this study, we aimed to elucidate the effect of propofol on H_2_O_2_-treated myocardial cells and rats with MIRI. Oxidative markers and cell apoptosis were analyzed to evaluate cardiomyocyte injury, and myocardial infarction in rats was measured to assess MIRI. We found that propofol inhibited myocardial damage, oxidative stress, and apoptosis of H_2_O_2_-treated H9c2 cells, and reduced myocardial infarction in MIRI rats by regulating the GSK3β-Nrf2/HO-1 signaling pathway. These findings provide new insights into the treatment of ischemic heart disease.

### 3.1. The effects of propofol on H9c2 cells

To determine the appropriate propofol concentration, H9c2 cells were treated with different concentrations (0, 50, 100, and 200 μM). Figure 1(a) shows the structure of propofol. The viability of H9c2 cells showed no significant differences between the 0, 50, and 100 μM groups, but remarkably decreased in cells treated with 200 μM propofol (Figure 1(b)). Therefore, cells were treated with 50 μM propofol for the L-PRO group and 100 μM propofol for the H-PRO group.

**Figure 1.** Effect of propofol on H9c2 cell viability.

(a) The molecular structure of propofol. (b) Cell viability from three replicates of H9c2 cells was analyzed using the Cell Counting Kit-8 assay. *P < 0.01 vs. CON group.

### 3.2. Propofol suppressed H_2_O_2_-induced cardiomyocyte injury and oxidative stress in H9c2 cells

As shown in Figure 2(a-f), H_2_O_2_ exposure markedly increased the levels of CK-MB, cTn-1, LDH, MDA, and CAT, and decreased the levels of GSH, SOD, and ROS. However, propofol treatment significantly decreased the levels of CK-MB, cTn-1, LDH, MDA, and CAT, and increased the levels of GSH, SOD, and ROS in H_2_O_2_-treated cells in a dose-dependent manner.

**Figure 2.** Effect of propofol on cardiomyocyte injury and oxidative stress of H_2_O_2_-treated H9c2 cells.

The levels of (a) creatine kinase-MB (CK-MB) and (b) cardiac troponin-1 (cTn-1) were determined using enzyme-linked immunosorbent assays (ELISAs). (c) Lactate dehydrogenase (LDH), (d) glutathione (GSH), (e) superoxide dismutase (SOD), (f) malondialdehyde (MDA), (g) reactive oxygen species (ROS), and (h) catalase (CAT) levels were measured in H9c2 cells treated with H_2_O_2_ and low- or high-dose propofol using corresponding kits. Experiments were performed in triplicate. ***P < 0.001, **P < 0.01 vs. CON group. ^###^*P* < 0.001, ^##^*P* < 0.01, and ^#^*P* < 0.05 vs. H_2_O_2_ group.

### 3.3. Propofol suppressed the apoptosis of H9c2 cells

We determined the effect of propofol on apoptosis in H9c2 cells using TUNEL assays and flow cytometry. The rate of apoptosis was significantly higher in the H_2_O_2_ group than the CON group. Propofol substantially decreased the rate of apoptosis of H_2_O_2_-treated H9c2 cells (Figure 3(a,b)). Moreover, propofol increased the mRNA and protein expression levels of Bcl-2 and decreased the levels of BAX (Figure 3(c,d)).

**Figure 3.** Effect of propofol on the apoptosis of H_2_O_2_-treated H9c2 cells.

(a) Flow cytometry was performed to evaluate apoptosis, and the apoptosis rate was quantified. (b) TUNEL assays were performed to assess apoptosis and TUNEL-positive cells were quantified. (c) The mRNA expression levels of *Bax* and *Bcl-2* were analyzed using quantitative reverse transcription-polymerase chain reaction (qRT-PCR). (d) The protein levels of Bax and Bcl-2 were determined using Western blotting. All experiments were performed in triplicate. ***P < 0.001, **P < 0.01 vs. CON group. ^#^*P* < 0.05, ^##^*P* < 0.01 vs. H_2_O_2_ group.

### 3.4. Propofol alleviated myocardial infarction in rats

We determined the effect of propofol on myocardial infarction in rats. Compared to the sham group, the MIRI group exhibited significant myocardial infarction. Meanwhile, propofol substantially decreased the infarction area in the hearts of rats with MIRI (Figure 4(a,b)).

**Figure 4.** Effect of propofol on MIRI *in vivo.*

(a) Myocardial infarction was evaluated using Evans blue dye staining. (b) The areas of myocardial infarction from five rats were quantified. ***P < 0.001 vs. sham group. ^##^*P* < 0.01 vs. H_2_O_2_ group.

### 3.5. Propofol upregulated the GSK3β-Nrf2/HO-1 signaling pathway in H9c2 cells

We tested the effect of propofol on the GSK3β-Nrf2/HO-1 signaling pathway in H9c2 cells. As shown in Figure 5(a,b), propofol treatment significantly increased the mRNA expression levels of *Nrf2* and *HO-1* in H_2_O_2_-treated cells, while it markedly increased the protein expression levels of Nrf2, HO-1, and NQO1; decreased the levels of p-GSK3β and p-Fyn; but did not affect the levels of GSK3β or Fyn (Figure 5(c)). Moreover, nuclear Nrf2 levels were increased by propofol in H_2_O_2_-treated cells, but the localization of Nrf2 in the cytoplasm was almost unaffected by H_2_O_2_ or propofol (Figure 6((a-c)). Propofol treatment induced the upregulation of Nrf2 and HO-1 in a time-dependent manner (Figure 7(a-c)).

**Figure 5.** Effect of propofol on the GSK3β-Nrf2/HO-1 signaling pathway.

The mRNA expression levels of (a) *Nrf2* and (b) *HO-1* were determined using qRT-PCR. (c) The protein expression levels of Nrf2, HO-1, p-GSK3β, GSK3β, p-Fyn, Fyn, and NQO1 were measured using Western blotting. All experiments were performed in triplicate. ***P < 0.001, **P < 0.01 vs. CON group. ^###^*P* < 0.001, ^##^*P* < 0.01, and ^#^*P* < 0.05 vs. H_2_O_2_ group.

**Figure 6.** Effect of propofol on Nrf2 localization in the nucleus and cytoplasm.

(a-c) The localization of Nrf2 in the nucleus and cytoplasm was detected using Western blotting. ***P < 0.001 vs. CON group. ^##^*P* < 0.01, and ^#^*P* < 0.05 vs. H_2_O_2_ group.

**Figure 7.** Effect of propofol on Nrf2 and HO-1 expression levels.

(a-c) After propofol treatment for 0, 12, 24, and 48 h, the protein expression levels of Nrf2 and HO-1 were measured using Western blotting. ***P < 0.001 vs. CON group. ^###^*P* < 0.001, ^##^ *P* < 0.01, and ^#^*P* < 0.05 vs. 0 h group.

### 3.6. Nrf2 knockdown induced the degradation of H9c2 cells

To further verify the potential role of Nrf2 signaling in cardiomyocyte injury, rescue assays were performed. As shown in Figure 8(a-h), knockdown of Nrf2 significantly alleviated the effects of propofol and induced the degradation of cardiomyocytes, as manifested by the exacerbation of cardiomyocyte injury and oxidative stress. Moreover, knockdown of Nrf2 promoted the apoptosis of H9c2 cells (Figure 9(a-c)). Additionally, silencing of Nrf2 blocked the mRNA and/or protein expression of BAX and Bcl-2 and inactivated the GSK3β/Nrf2/HO-1 signaling pathway (Figure 10(a,b)).

**Figure 8.** Effect of Nrf2 knockdown on H_2_O_2_-induced cardiomyocyte injury and oxidative stress.

The levels of (a) CK-MB and (b) cTn-1 were determined using ELISAs. (c) LDH, (d) GSH, (e) SOD, (f) MDA, (g) ROS, and (h) CAT levels in H9c2 cells were measured using corresponding kits following the knockdown of Nrf2. All experiments performed in triplicate. ***P < 0.001, **P < 0.01 vs. CON group. ^##^*P* < 0.01, ^#^*P* < 0.05 vs. H_2_O_2_ + propofol + sh-NC group.

**Figure 9.** Effect of Nrf2 knockdown on the apoptosis rates of H9c2 cells.

(a) The expression of *Nrf2* following shRNA transfection was determined using qRT-PCR. (b) Flow cytometry was performed to measure the apoptosis rate of H9c2 cells. (c) Apoptosis was evaluated using the TUNEL staining assay. All experiments were performed in triplicate. **P < 0.01 vs. sh-NC group. ***P < 0.001 vs. CON group. ^##^*P* < 0.01, ^#^*P* < 0.05 vs. H_2_O_2_ + propofol + sh-NC group.

**Figure 10.** Effect of Nrf2 knockdown on apoptosis-related factors and the GSK3β-Nrf2/HO-1 signaling pathway.

(a) The mRNA expression levels of *Bax, Bcl-2, Nrf2*, and *HO-1* were determined using qRT-PCR. (b) The protein levels of Bax, Bcl-2, Nrf2, HO-1, p-GSK3β, and GSK3β were determined using Western blotting. All experiments were performed in triplicate. ***P < 0.001, **P < 0.01 vs. CON group. ^##^*P* < 0.01, ^#^*P* < 0.05 vs. H_2_O_2_ + propofol + sh-NC group.

## 4. Discussion

The present study revealed that treating MIRI requires a greater understanding of its pathophysiological process. Identifying novel signaling pathways that can be targeted by small molecules is important for developing new treatments. In this study, we found that propofol ameliorated the H_2_O_2_-induced injury of H9c2 cells by downregulating the GSK3β-Nrf2/HO-1 signaling pathway. In addition, we found that treating rats with MIRI with propofol significantly reduced the myocardial infarction size. Our observations suggested that the effect of propofol may be standardized to modulate the GSK3β-Nrf2/HO-1 signaling pathway before myocardial reperfusion. However, the knockdown of Nrf2 promoted cardiomyocyte apoptosis and the oxidative stress response, which further induced MIRI.

The protective effect of propofol against myocardial infarction has been linked to its anti-apoptotic [26] and antioxidant [27,28] effects. The GSK3β-Nrf2/HO-1 signaling pathway has been implicated in oxidative stress regulation and apoptosis [29, 30]. Accumulating evidence shows that propofol alleviates oxidative stress in myocardial cells and in injured liver, kidney, and lung tissue by activating the Nrf2/HO-1 pathway [31–34]. However, most previous studies have only focused on the effect of propofol on the Nrf2/HO-1 pathway. In the present study, we examined the effect of propofol on apoptosis. A previous study reported that propofol is related to tumor cell apoptosis [35]. We found that propofol reduced the incidence of myocardial infarction in rats with MIRI and suppressed oxidative stress and apoptosis in H_2_O_2_-treated H9c2 cells, which was consistent with the results of previous studies [36–38]. Additionally, propofol has been shown to interfere with the cardioprotective effects of remote ischemic conditioning [39], which is inconsistent with our findings. Currently, the mechanism responsible for the inhibitory effects of propofol on remote ischemic preconditioning remains unclear. However, it may be due to propofol decreasing STAT5 phosphorylation, inactivating sensory fibers, or disrupting vagal nerve control. Thus, the reported roles of propofol in myocardial protection are contradictory, and it is necessary to provide more information to allow the appropriate clinical application of propofol.

The complexity of the MIRI process led us to explore a novel signaling pathway that may be a viable target of propofol, confirming it as a feasible hallmark in the treatment of MIRI. The involvement of the GSK3β-Nrf2-HO-1 pathway in the MIRI process has previously been reported [5,10,11]. Nrf2 is a key regulator of oxidative stress induced by cell death, such as apoptosis, ferroptosis, and pyroptosis. As a transcription factor, Nrf2 activates iron and oxidative signaling. For instance, Nrf2 interacts with Pitx2 to repair heart function by stimulating antioxidant signaling [40]. However, the dysfunction of Nrf2 induces excessive cardiac oxidative stress, senescence, and cell death [41,42]. Therefore, the activation of Nrf2 signaling may play a beneficial role in the treatment of heart disease. In this study, propofol was found to significantly increase the gene expression levels of *Nrf2, HO-1*, and *Bcl-2*, while inhibiting *Bax* gene expression levels. The effect of propofol on Nrf2 was mainly to increase its localization in the nucleus. However, Nrf2 knockdown interfered with the cellular function of cardiomyocytes. Thus, we postulate that the effect of propofol is associated with many other antioxidants that have been shown to regulate genes such as Bax and Bcl-2 [43].

However, this study has some limitations that should be noted. The study mainly focused on the effect of propofol on myocardial cell injury *in vitro* and few experiments were performed on rats with MIRI. Our future studies will explore the role of propofol in rats with MIRI and translate our findings into clinical applications. Moreover, we will investigate whether the effect of propofol is due only to its antioxidant properties or whether it also involves other mechanisms.

## 5. Conclusions

Propofol attenuated H_2_O_2_-induced myocardial cell injury *in vitro* and protected against MIRI in rats. Mechanistically, propofol exerted its effects on cells by modulating the GSK3β-Nrf2/HO-1 signaling pathway. These findings suggested that propofol may be a promising agent for treating MIRI.

## Data Availability

The authors confirm that the data supporting the findings of this study are available within the article.

## Research highlights

1. Propofol alleviated injury in H_2_O_2_-treated H9c2 cells.
2. Propofol alleviated oxidative stress and apoptosis of H_2_O_2_-treated H9c2 cells.
3. Propofol decreased myocardial infarction in rats with MIRI.
4. Propofol activated the GSK3β/Nrf2/HO-1 signaling pathway.
5. Propofol alleviated cardiomyocyte injury by activating the GSK3β/Nrf2/HO-1 pathway.

## References

[1] Severino P, D’Amato A, Pucci M, et al. Ischemic heart disease pathophysiology paradigms overview: from plaque activation to microvascular dysfunction. Int J Mol Sci. 2020;21(21):8118.10.3390/ijms21218118PMC766325833143256

[2] Lapointe-Shaw L, Bell CM. Acute myocardial infarction. Bmj. 2014;348(jan21 5):f7696–f7696.2445240710.1136/bmj.f7696

[3] Amani H, Habibey R, Hajmiresmail SJ, et al. Antioxidant nanomaterials in advanced diagnoses and treatments of ischemia reperfusion injuries. J Mater Chem B. 2017;5(48):9452–9476.3226456010.1039/c7tb01689a

[4] Ueda K, Takano H, Niitsuma Y, et al. Sonic hedgehog is a critical mediator of erythropoietin-induced cardiac protection in mice. J Clin Invest. 2010;120(6):2016–2029.2048481210.1172/JCI39896PMC2877931

[5] Liu CW, Yang F, Cheng SZ, et al. Rosuvastatin postconditioning protects isolated hearts against ischemia-reperfusion injury: the role of radical oxygen species, PI3K-Akt-GSK-3beta pathway, and mitochondrial permeability transition pore. Cardiovasc Ther. 2017;35(1):3–9.2758001710.1111/1755-5922.12225

[6] Jacobs KM, Bhave SR, Ferraro DJ, et al. GSK-3beta: a bifunctional role in cell death pathways. Int J Cell Biol. 2012;2012:930710.2267536310.1155/2012/930710PMC3364548

[7] Li C, Pan Z, Xu T, et al. Puerarin induces the upregulation of glutathione levels and nuclear translocation of Nrf2 through PI3K/Akt/GSK-3*β* signaling events in PC12 cells exposed to lead. Neurotoxicol Teratol. 2014;46:1–9.2519571710.1016/j.ntt.2014.08.007

[8] Alam J, Stewart D, Touchard C, et al. Nrf2, a Cap’n’Collar transcription factor, regulates induction of the heme oxygenase-1 gene. J Biol Chem. 1999;274(37):26071–26078.1047355510.1074/jbc.274.37.26071

[9] Zhang X, Yu Y, Lei H, et al. The Nrf-2/HO-1 signaling axis: a ray of hope in cardiovascular diseases. Cardiol Res Pract. 2020;2020:5695723.3241144610.1155/2020/5695723PMC7204387

[10] Bonnefont-Rousselot D. Resveratrol and cardiovascular diseases. Nutrients. 2016;8(5):250.10.3390/nu8050250PMC488266327144581

[11] Liu X, Wei J, Peng DH, et al. Absence of heme oxygenase-1 exacerbates myocardial ischemia/reperfusion injury in diabetic mice. Diabetes. 2005;54(3):778–784.1573485610.2337/diabetes.54.3.778

[12] Naito H, Nojima T, Fujisaki N, et al. Therapeutic strategies for ischemia reperfusion injury in emergency medicine. Acute Med Surg. 2020;7(1):e501–n/a.10.1002/ams2.501PMC723156832431842

[13] Bryson HM, Fulton BR, Faulds D. Propofol: an update of its use in anaesthesia and conscious sedation. Drugs. 1995;50(3):513–559. (New York, N.Y.).852177210.2165/00003495-199550030-00008

[14] Kato R, Foex P. Myocardial protection by anesthetic agents against ischemia-reperfusion injury: an update for anesthesiologists. Can J Anaesth. 2002;49(8):777–791.1237470510.1007/BF03017409

[15] Gao X, Mi Y, Guo N, et al. The mechanism of propofol in cancer development: an updated review. Asia Pac J Clin Oncol. 2020;16(2):e3–e11.3197093610.1111/ajco.13301

[16] Romuk EB, Szczurek W, Nowak PG, et al. Effects of propofol on the liver oxidative-antioxidant balance in a rat model of Parkinson’s disease. Adv Clin Exp Med. 2016;25(5):815–820.2802894210.17219/acem/36459

[17] Searle NR, Sahab P. Propofol in patients with cardiac disease. Can J Anaesth. 1993;40(8):730–747.840315810.1007/BF03009770

[18] Ko SH, Yu CW, Lee SK, et al. Propofol attenuates ischemia-reperfusion injury in the isolated rat heart. Anesth Analg. 1997;85(4):719–724.932244510.1097/00000539-199710000-00002

[19] Kokita N, Hara A. Propofol attenuates hydrogen peroxide-induced mechanical and metabolic derangements in the isolated rat heart. Anesthesiology. 1996;84(1):117–127.857232410.1097/00000542-199601000-00014

[20] Chen X, Wang Y, Xiao ZY, et al. Effect of propofol on myocardial ischemia/reperfusion injury in rats through JAK/STAT signaling pathway. Eur Rev Med Pharmacol Sci. 2019;23(14):6330–6338.3136414010.26355/eurrev_201907_18456

[21] Yan HJ, Qi GQ, Ma Y. Effect of propofol on myocardial ischemia-reperfusion injury through MAPK/ERK pathway. Eur Rev Med Pharmacol Sci. 2019;23(24):11051–11061.3185857710.26355/eurrev_201912_19813

[22] Jin Z, Wang WF, Huang JP, et al. Dryocrassin ABBA induces apoptosis in human hepatocellular carcinoma HepG2 cells through a caspase-dependent mitochondrial pathway. Asian Pac J Cancer Prev. 2016;17(4):1823–1828.2722185910.7314/apjcp.2016.17.4.1823

[23] Zhang B, Zhai M, Li B, et al. Honokiol ameliorates myocardial ischemia/reperfusion injury in type 1 diabetic rats by reducing oxidative stress and apoptosis through activating the SIRT1-Nrf2 signaling pathway. Oxid Med Cell Longev. 2018;2018:3159801.2967513210.1155/2018/3159801PMC5838504

[24] Fei L, Zhang J, Niu H, et al. Effects of rosuvastatin and MiR-126 on myocardial injury induced by acute myocardial infarction in rats: role of Vascular Endothelial Growth Factor A (VEGF-A). Med Sci Monit. 2016;22:2324–2334.2737640510.12659/MSM.896983PMC4941889

[25] Zhou D, Zhuang J, Wang Y, et al. Propofol alleviates DNA damage induced by oxygen glucose deprivation and reperfusion via FoxO1 nuclear translocation in H9c2 cells. Front Physiol. 2019;10:223.3093079010.3389/fphys.2019.00223PMC6429026

[26] Jin YC, Kim W, Ha YM, et al. Propofol limits rat myocardial ischemia and reperfusion injury with an associated reduction in apoptotic cell death in vivo. Vascul Pharmacol. 2009;50(1–2):71–77.1899622410.1016/j.vph.2008.10.002

[27] Adaramoye OA, Akinwonmi O, Akanni O. Effects of propofol, a sedative-hypnotic drug, on the lipid profile, antioxidant indices, and cardiovascular marker enzymes in wistar rats. ISRN Pharmacol. 2013;2013:230261.10.1155/2013/230261PMC369063423840962

[28] Murphy PG, Myers DS, Davies MJ, et al. The antioxidant potential of propofol (2,6-diisopropylphenol). Br J Anaesth. 1992;68(6):613–618.131918910.1093/bja/68.6.613

[29] Habtemariam S, Mario Z, Zoratti M. The Nrf2/HO-1 axis as targets for flavanones: neuroprotection by pinocembrin, naringenin, and eriodictyol. Oxid Med Cell Longev. 2019;2019:4724920.3181487810.1155/2019/4724920PMC6878820

[30] Yan C, Zhang X, Miao J, et al. Farrerol directly targets GSK-3beta to activate Nrf2-ARE pathway and protect EA.hy926 cells against oxidative stress-induced injuries. Oxid Med Cell Longev. 2020;2020: 5967434.10.1155/2020/5967434PMC700795032082480

[31] Ge M, Chen H, Zhu Q, et al. Propofol post-conditioning alleviates hepatic ischaemia reperfusion injury via BRG1-mediated Nrf2/HO-1 transcriptional activation in human and mice. J Cell Mol Med. 2017;21(12):3693–3704.2874900810.1111/jcmm.13279PMC5706583

[32] Ge M, Luo G, Yao W, et al. Propofol pretreatment attenuates remote kidney injury induced by orthotopic liver autotransplantation, which is correlated with the activation of Nrf2 in rats. Mol Med Rep. 2015;11(5):3962–3968.2552950810.3892/mmr.2014.3126

[33] Kamada N, Kanaya N, Hirata N, et al. Cardioprotective effects of propofol in isolated ischemia-reperfused Guinea pig hearts: role of KATP channels and GSK-3beta. Can J Anaesth. 2008;55(9):595–605.1884058910.1007/BF03021433

[34] Yao W, Luo G, Zhu G, et al. Propofol activation of the Nrf2 pathway is associated with amelioration of acute lung injury in a rat liver transplantation model. Oxid Med Cell Longev. 2014;2014:258567.2466928210.1155/2014/258567PMC3941594

[35] Li Z, Liu H, Zhang Y, et al. The effect of propofol on the proliferation and apoptosis of hepatocellular carcinoma cells through TGF-beta1/Smad2 signaling pathway. Bioengineered. 2021;12(1):4581–4592.3432364710.1080/21655979.2021.1955177PMC8806409

[36] Engelhard K, Werner C, Eberspacher E, et al. Influence of propofol on neuronal damage and apoptotic factors after incomplete cerebral ischemia and reperfusion in rats: a long-term observation. Anesthesiology. 2004;101(4):912–917.1544852410.1097/00000542-200410000-00016

[37] Runzer TD, Ansley DM, Godin DV, et al. Tissue antioxidant capacity during anesthesia: propofol enhances in vivo red cell and tissue antioxidant capacity in a rat model. Anesth Analg. 2002;94(1):89–93. table of contents.1177280710.1097/00000539-200201000-00017

[38] Xia Z, Godin DV, Chang TK, et al. Dose-dependent protection of cardiac function by propofol during ischemia and early reperfusion in rats: effects on 15-F2t-isoprostane formation. Can J Physiol Pharmacol. 2003;81(1):14–21.1266525310.1139/y02-170

[39] Heusch G. Remote ischemic conditioning in cardiovascular surgery. J Cardiovasc Pharmacol Ther. 2017;22(4):297–301.2858758010.1177/1074248416687874

[40] Tao G, Kahr PC, Morikawa Y, et al. Pitx2 promotes heart repair by activating the antioxidant response after cardiac injury. Nature. 2016;534(7605):119–123.2725128810.1038/nature17959PMC4999251

[41] Chen K, Wang S, Sun QW, et al. Klotho deficiency causes heart aging via impairing the Nrf2-GR pathway. Circ Res. 2021 Feb 19;128(4):492–507.3333412210.1161/CIRCRESAHA.120.317348PMC8782577

[42] Xu S, Wu B, Zhong B, et al. Naringenin alleviates myocardial ischemia/reperfusion injury by regulating the nuclear factor-erythroid factor 2-related factor 2 (Nrf2) /System xc-/ glutathione peroxidase 4 (GPX4) axis to inhibit ferroptosis. Bioengineered. 2021;12(2):10924–10934.3469931710.1080/21655979.2021.1995994PMC8809912

[43] Lee YS, Kang YJ, Kim HJ, et al. Higenamine reduces apoptotic cell death by induction of heme oxygenase-1 in rat myocardial ischemia-reperfusion injury. Apoptosis. 2006;11(7):1091–1100.1670326410.1007/s10495-006-7110-y

